# Motor Function Assessment of Upper Limb in Stroke Patients

**DOI:** 10.1155/2021/6621950

**Published:** 2021-02-24

**Authors:** Bingyu Pan, Zhen Huang, Tingting Jin, Jiankang Wu, Zhiqiang Zhang, Yanfei Shen

**Affiliations:** ^1^School of Sports Engineering, Beijing Sport University, Beijing, China; ^2^Rehabilitation Department, Peking University First Hospital, Beijing, China; ^3^Sensor Network and Application Research Centre, School of Electronic Electrical and Communication Engineering, University of Chinese Academy of Sciences, Beijing, China; ^4^School of Electronic and Electrical Engineering, University of Leeds, Leeds, UK

## Abstract

**Background:**

Quantitative assessment of motor function is extremely important for poststroke patients as it can be used to develop personalized treatment strategies. This study aimed to propose an evaluation method for upper limb motor function in stroke patients.

**Methods:**

Thirty-four stroke survivors and twenty-five age-matched healthy volunteers as the control group were recruited for this study. Inertial sensor data and surface electromyography (sEMG) signals were collected from the upper limb during voluntary upward reaching. Five features included max shoulder joint angle, peak and average speeds, torso balance calculated from inertial sensor data, and muscle synergy similarity extracted from sEMG data by the nonnegative matrix factorization algorithm. Meanwhile, the Fugl–Meyer score of each patient was graded by professional rehabilitation therapist.

**Results:**

Statistically significant differences were observed among severe, mild-to-moderate, and control group of five features (*p* ≤ 0.001). The features varied as the level of upper limb motor function changes since these features significantly correlated with the Fugl–Meyer assessment scale (*p* ≤ 0.001). Moreover, the Bland–Altman method was conducted and showed high consistency between the evaluation method of five features and Fugl–Meyer scale. Therefore, the five features proposed in this paper can quantitatively evaluate the motor function of stroke patients which is very useful in the rehabilitation process.

## 1. Introduction

Stroke is a global disease with high mortality and high disability caused by motor cortical damage [1]. According to the statistics, there were approximately 13.68 million new increased stroke patients worldwide a year and about 70% of survivors had different degrees of upper limb and hand movement dysfunction [2]. The recovery of patients' motor function mainly depends on rehabilitation training. However, due to individual difference of patients, it is critical to generate personalized rehabilitation program according to the different motor impairment levels.

Thus far, medical scale methods have been widely used in clinics to evaluate motor functions of stroke patients, including Brunnstrom approach [3, 4], Fugl–Meyer (FM) assessment scale [5], Motor Assessment Scale (MAS) [6], and Wolf Motor Function Test (WMF) [7]. Among them, FM assessment is currently recognized and the most widely used clinical evaluation method [8]. The FM scale was developed based on Brunnstrom approach, where patients completed a series of motions following instructions, and scored by physicians according to the completion degree of the movements [9]. Although the medical scales have good reliability and validity, the results relied on subjective scores from physicians and difficult to reflect minor functional changes due to rough evaluation. Some poststroke patients may have the same evaluation score but with different movement performance. Thus, it would be helpful to develop a quantitative evaluation method with respect to the specific motion of poststroke patients that can reveal the patients' deficits and provide advice on the rehabilitation process.

In recent years, inertial sensors have been applied to monitor human movement and are widely used because of their low price. There is a debate about the correlation between clinical scales and kinematic parameters in poststroke patients. Yu et al. applied the accelerometer signals obtained from the wearable sensor network to establish the Brunnstrom stage classification, which classified patients into six stages according to the degree of recovery [10]. Zhang et al. extracted mathematical features from raw kinetic data, such as maximum magnitude of raw data to implement automatic Brunnstrom stage classification for upper-extremity rehabilitation [11]. However, these studies gave roughly stage of motor impairment since the Brunnstrom scale only had six stages and the features proposed cannot provide much information about how the movement was completed. The relationship between FM scores and kinematic measures was also studied [12, 13], but neural deficits may be ignored at the kinematic level as similar movements can be produced through different neuromuscular mechanisms. Recent advances have been made in the use of the surface electromyography (sEMG)-based motion evaluation method. sEMG factorization procedures are used to facilitate the analysis of complex muscle activation patterns. For example, matrix factorization techniques attempt to model complex multivariate data as linear combinations of a small set of basis vectors [14]. The central nervous system (CNS) simplifies the control of motor tasks by using a low-dimensional modular organization of muscle activation, which is called muscle synergy [15]. The concept of muscle synergy was first proposed by scholar Bernstein and became the theoretical basis for redundant control problems in the CNS [16]. Muscle synergies have been identified as building blocks for a variety of motor tasks in humans [17]. Muscle synergy is a relatively new concept in neurorehabilitation, which can offer clinicians insight into underlying neural strategies [18]. Muscle synergies reflect the injury of the cerebrovascular accident and could document the effects of the functional recovery due to a suitable and customized treatment [19]. Cheung et al. found that the recruitment patterns of muscle synergies may alter in stroke patients [20]. Studies have found that spinal cord stimulation influences motor function through muscle synergy activation after injury [21]. Ji et al. used the muscle synergy method to quantify the characteristics that underlie ankle muscle activation [22]. Yang et al. found temporal features of muscle synergies in sit-to-stand motion reflecting the motor impairment of poststroke patients [23]. Moreover, Shuman et al. observed that cerebral palsy children whose synergy activations were more similar to typically developing peers after treatment had greater improvements in gait [24]. Although there are many studies regarding muscle synergies in poststroke locomotion, the quantitative measurement of muscle synergy in reaching movement of stroke patients is still unsolved.

Motor function assessment of the upper limb in stroke patients was studied in this paper. The proposed five features could provide relatively comprehensive information about the completion of movements. This information is important for therapists to conduct personalized rehabilitation therapy for stroke patients. Special training can be developed based on the results to make patients' features more similar to the control.

## 2. Materials and Methods

### 2.1. Experimental Protocol

Thirty-four stroke survivors and twenty-five age-matched healthy adults serving as the control group were recruited from the Peking University First Hospital for this study. All the stroke participants for our research were diagnosed with stroke for the first time, poststroke duration no longer than six months and shoulder could lift at least 30° without help. Moreover, patients were not with other musculoskeletal disease. The Fugl–Meyer score of each patient was graded by professional rehabilitation therapist. We only used the FM score of the upper limb (without hand) since we focused on the evaluation of upper limb motor function. The patients were classified into two groups according to their FM score, severe impaired (FM ≤ 30) and mild-to-moderate impaired (FM > 30) [25]. As a result, 19 of 34 patients were mild-to-moderate impaired and 15 patients were severe impaired. The general information of participants is shown in Table 1. This research has been approved by the Ethics Committee of Peking University First Hospital, and all the participants gave informed consent before experiments.

When the experiment started, the subject sat upright in front of an appropriate table and was asked to reach for the objects placed on the table by the movement of upward reaching and then held on for 2 seconds at the highest point. The object for reaching was placed at the point where subjects could reach it by shoulder flexion of 90° while forearm supination was 0° (thumbs up).

### 2.2. Data Acquisition and Preprocessing

The kinematic data were recorded (50 Hz) by the wireless upper limb motion capture system consisting of four MPU-9150 (InvenSense Inc, Sunnyvale, USA) inertial measurement units (IMU), which were attached to the middle of the waist, upper arm, forearm, and hand, respectively. Each sensor included a triaxial accelerometer, triaxial gyroscope, and triaxial magnetometer. sEMG activity of 7 muscles wrapping across shoulder, upper arm, and forearm was synchronously recorded (1000 Hz) by the ME6000 multichannel bipolar sEMG recording system (Mega Electronics Ltd, Kuopio, Northern Savonia, Finland). The recorded muscles were pectoralis major (PECM), trapezius (TRA), anterior deltoid (DELA), medial deltoid (DELM), biceps brachii (BIC), triceps brachii (TRI), and brachioradialis (BRAC). Electrodes were placed on corresponding muscles consistent with the recommendations of the Surface Electromyography for the Noninvasive Assessment of Muscles (SENIAM) [26]. The IMU and sEMG sensors were attached to the affected side for stroke patients and dominant arm for healthy controls. Both the kinematic data and sEMG data were collected at the same time when subjects performed the movements. Diagram of data collection and sensor placement is shown in Figure 1.

Before muscle synergy analysis, the collected sEMG signals needed to be preprocessed first. sEMG signals were filtered with a high-pass, window-based finite impulse response filter with the cut-off of 50 Hz, then rectified and filtered by a low-pass window-based finite impulse response filter with the cut-off of 20 Hz, and finally integrated over 20 ms intervals to extract the envelope of sEMG signals and keep synchronous with the kinematic data. The sEMG signals from each muscle of each arm were normalized by maximum value to facilitate comparisons between muscles and subjects.

All data were saved and then analyzed with Matlab 2017a (the Mathworks, Natick, USA).

## 3. Evaluation Features

### 3.1. Max Shoulder Joint Angle

Max shoulder joint angle which represents the shoulder range of motion can be used to directly demonstrate the completeness of a task. With real-time shoulder joint angle, the upper limb trajectory can be reconstructed and can provide information about the quality of a specific task. The upper limb joint angle is obtained on the basis of the hierarchical biomechanical model [27, 28]. To calculate shoulder joint angles, we assume that upper arm, forearm, and hand are all rigid bodies, rotating around their corresponding joints. The quaternions are obtained by fusing data of accelerometer, gyroscope, and magnetometer from inertial sensors according to previous studies [28]:

(1) $$\begin{array}{c} q_{o}^{BS}={\left(q_{o}^{GB}\right)}^{-1}\cdot q_{o}^{GS},\\ q_{t}^{GB}=q_{t}^{GS}\cdot q_{t}^{SB}=q_{t}^{GS}\cdot {\left(q_{t}^{BS}\right)}^{-1}, \end{array}$$

where the superscript *G* means the global, *B* means the body, and *S* means the sensor. The subscript *o* means the initial of time and *t* means at time *t*. So, *q*_*o*_^*GB*^ is the quaternion of the body in global coordinates in the initial. *q*_*o*_^*BS*^ remains the same at different time, which means *q*_*t*_^*BS*^=*q*_*o*_^*BS*^. Then, the position vector *P*_elbow_ of elbow joint is calculated by the following:

(2) $$\begin{array}{c} \;P_{\text{elbow}}^{G}=P_{\text{shoulder}}^{G}+q_{\text{shoulder}}^{GB}⊗\;L_{\text{upper}}^{B}⊗\;{\left(q_{\text{shoulder}}^{GB}\right)}^{-1}, \end{array}$$

where *L*_upper_^*B*^ is the vector of the upper limb in the body coordination system. In this case, shoulder joint angle is equal to the angle between upper limb vectors of start point to endpoint [27]:

(3) $$\begin{array}{c} \theta =\;\cos^{-1}P_{\text{elbow}}^{s},P_{\text{elbow}}^{e}, \end{array}$$

where *P*_elbow_^*s*^ and *P*_elbow_^*e*^ are the start point and endpoint of elbow joint, respectively. Equation (4) can be simplified as follows:

(4) $$\begin{array}{c} \theta =\;\cos^{-1}\langle \begin{array}{c} q_{\text{shoulder}}^{s}⊗L_{\text{upper}}^{B}⊗{\left(q_{\text{shoulder}}^{s}\right)}^{-1}\\ q_{\text{shoulder}}^{e}⊗L_{\text{upper}}^{B}⊗{\left(q_{\text{shoulder}}^{e}\right)}^{-1} \end{array}\rangle , \end{array}$$

where *q*_shoulder_^*s*^ and *q*_shoulder_^*e*^ are the start point and endpoint of shoulder quaternion, respectively. The max shoulder joint angle is the max value during the upward reaching movement, and to avoid the sudden extreme value, we take the mean value within a short window (5 points) and calculate the maximum value.

### 3.2. Upper Arm Peak Speed

In clinical practice, stroke patients' multijoint pointing movements are characterized by decreased movement speed and increased movement variability with respect to healthy subjects [29]. Therefore, we calculate instantaneous speed objectively and quantitatively by the first-order differential of the joint position. Peak speed is the maximal instantaneous speed throughout the reaching movement, where the instantaneous speed is given as follows:

(5) $$\begin{array}{c} v\left(i\right)=\frac{1}{\Delta t}\sqrt{{\left(\left.P_{x}^{i+1}-P_{x}^{i}\right)\right)}^{2}+{\left(P_{y}^{i+1}-P_{y}^{i}\right)}^{2}+{\left(P_{z}^{i+1}-P_{z}^{i}\right)}^{2}}, \end{array}$$

in which Δ*t* is the sampling interval and *P*_*x*_^*i*^,  *P*_*y*_^*i*^,  and *P*_*z*_^*i*^ are the three-dimensional coordinates at sampling moment of *i*, which can be obtained by equation (2). The peak speed we used here is the maximum value of instantaneous speed, and to avoid the sudden extreme value, we take the mean value within a short window (5 points) and calculate the maximum value.

### 3.3. Upper Arm Average Speed

The average speed of the upper arm is the average speed at which the subject completes the entire movement of reaching, reflecting the efficiency of completing the task. The average is calculated by the mean value of instantaneous speed obtained from equation (5).

### 3.4. Torso Balance Degree

Individuals with mild-to-moderate stroke have deficits in timing and spatial coordination of arm and torso movements during different parts of a reaching movement [30]. When performing the movement of reaching objects, stroke patients with limited arm movement can reach objects by using a compensatory strategy involving torso recruitment [31]. A similar strategy is observed in healthy individuals reaching for objects placed beyond the reach of the arm. The compensatory involvement of the torso is greater for patients with more severe motor deficits [32, 33]. Here, we use a quantitative description to measure the compensation of stroke survivors. Torso balance degree is the angle of the torso leaned forward during the movement. Therefore, the patient's torso compensatory condition can be reflected through the torso balance degree. The greater the value is, the more serious the patient's torso compensatory condition is. Torso balance is calculated as follows:

(6) $$\begin{array}{c} C_{\text{trunk}}=\frac{\max\left\{\left|\text{Roll}\left(\emptyset \right)\right|,\left|\text{Pitch}\left(\theta \right)\right|,\left|\text{Yaw}\left(\varphi \right)\right|\right\}}{90^{{}^{\circ}}}\cdot 100\%, \end{array}$$

where Roll(∅), Pitch(*θ*), and Yaw(*φ*) are the Euler angle converted by torso quaternion.

### 3.5. Similarity of Muscle Synergy

Muscle synergies are used by the motor system as a modular organization to simplify the control of movements [34]. Muscle synergy structure analysis may be a powerful tool to assess rehabilitation procedures [35]. We applied the nonnegative matrix factorization (NMF) algorithm to extract muscle synergy from sEMG data [36]. Muscle synergy hypothesis models the activity of muscles as a linear combination of time-invariant muscle synergies, each activated by a time-varying activation coefficient [37, 38]. This model is mathematically expressed as follows:

(7) $$\begin{array}{c} M\left(t\right)=\overset{N}{\underset{i=1}{\sum }}C_{i}\left(t\right)w_{i}+\varepsilon , \end{array}$$

where *M*(*t*) is the sEMG data at time *t, N* is the number of muscle synergies, *w*_*i*_ is the *i*th muscle synergy, *C*_*i*_(*t*) is the nonnegative activation vector for the *i*th synergy, and *ε* is the residual. To determine the minimum number of muscle synergies adequate to reconstruct each dataset, variance accounted for (VAF) is calculated.

(8) $$\begin{array}{c} \text{VAF}=100\times \left(1-\frac{\text{SSE}}{\text{SST}}\right)=1-\frac{\sum_{i=1}^{m}\sum_{j=1}^{t}{\left(M_{ij}-{\hat{M}}_{ij}\right)}^{2}}{\sum_{i=1}^{m}\sum_{j=1}^{t}{\left(M_{ij}\right)}^{2}}, \end{array}$$

where SSE is the sum of the squared residuals between reconstruction sEMG and original sEMG and SST is the sum of the squared sEMG data. We defined the minimum number of synergies required to achieve a mean VAF greater than 95% as the number of synergies underlying each dataset. We use the scalar product to measure the similarity between two muscle synergies. For two synergy metrics *W*=[*w*_1_, *w*_2_,…, *w*_*n*_1__] and *W*′=[*w*_1_′, *w*_2_′,…, *w*_*n*_2__′, ] (where *n*_1_and *n*_2_ are the numbers of synergies), the feature of synergy similarity (*S*_*W*_) is defined as follows:

(9) $$\begin{array}{c} S_{W}\left(W,W^{\prime }\right)=\frac{1}{n_{1}}\overset{n_{1}}{\underset{k=1}{\sum }}\max\left[{s\left(W_{k},W_{l}^{\prime }\right)|}_{l=1}^{n_{2}}\right], \end{array}$$

where *s*(*W*_*k*_, *W*_*l*_′) represents the similarity of *W*_*k*_ and *W*_*l*_′ calculated by scalar product.

Since different evaluation features (EFs) have different dimensions, for the sake of comparison, we use the min-max normalization method to normalize the evaluation features:

(10) $$\begin{array}{c} \bar{{\text{EF}}_{i}^{j}}=\frac{{\text{EF}}_{i}^{j}-\min\left\{{\text{EF}}_{1}^{j},\ldots ,{\text{EF}}_{n}^{j}\right\}}{\max\left\{{\text{EF}}_{1}^{j},\ldots ,{\text{EF}}_{n}^{j}\right\}-\min\left\{{\text{EF}}_{1}^{j},\ldots ,{\text{EF}}_{n}^{j}\right\}}. \end{array}$$

### 3.6. Statistics Methods

In this study, descriptive statistics include the calculation of the mean and standard deviation. One-way multivariate analysis of variance (MANOVA) is conducted to evaluate the intergroup differences of five proposed features. Two sample *T*-tests are used to analyze whether there existed difference in five proposed features between the severe, mild-moderate, and control group. To quantify the relationship between the features and motor function, we calculated the Spearman rank correlation coefficients between each feature and the FM score. Reported results were considered significant for *p* < 0.001.

## 4. Results and Analysis

### 4.1. Evaluation Feature Values in Severe, Mild-to-Moderate, and Control Groups

In order to explore the relationship between evaluation features and motor function, we analyze the five features in subjects with three types of motor function level.

We take one subject from severe, mild-to-moderate, and control group separately to show the real-time shoulder joint angle during reaching task in Figure 2. It can be seen that the severe patient has the lowest range of shoulder joint angle and most vibrant trend compared with the mild-to-moderate one and the control and takes longest time to arrive the peak range in reaching which means he has lowest speed of the upper arm. We can see that stroke patients usually have a narrower range of shoulder joint angle of the affected arm due to hemiplegia. Therefore, the max shoulder angle is used to measure the shoulder range of motion of each subject.

NMF was conducted to preprocessed sEMG signals of each participant to extract muscle synergies. The number of muscle synergies is shown as Figure 3. Typically, three synergies are adequate to reconstruct muscle activity during reaching task in both control and stroke groups by setting the VAF threshold of 95% a. Muscle synergy template of control, mild-to-moderate, and severe group is summarized as Figure 4, where distributions of muscle weights for three synergies are displayed across subjects in each group with the group mean and standard deviation. Compared with the control template, muscle synergy altered in stroke subjects and synergy patterns in the mild-to-moderate group are more similar to the control template. The first synergy in the control group is accounting for shoulder flexion by mainly activating DELA and DELM. The second and third synergies in the control group are dominated by activation of TRA and TRI, which are accounting for the torso stability and keeping the arm straight during the reaching movement. However, the increasing activation of PEMC, lack of activation of TRI, and abnormality of activation of TRA in both mild-to-moderate and severe group are the most striking differences compared with the control group.

We then calculate the values of the five features in three groups to preliminarily estimate the relationship between the features and the motor function level of the subjects. The result of MANOVA indicates significant differences of the five features in three groups (*p* = 9.39*E* − 06). The mean and standard error of mean of five features are shown as Figure 5. The asterisks in Figure 5 are used to denote those who have significant difference (*t*-test, *p* ≤ 0.001). The severe group is significantly different from mild-to-moderate and control groups, while the mild-to-moderate group is close to the control group. By comparison, there is a good agreement between the features and the motor function level of the subjects. The max shoulder angle, peak and average speeds, and muscle synergy similarity increased with the growth of motor function while the torso balance degree decreased, indicating that the more severe the loss of motor function, the lower the range of shoulder join, the lower peak speed, the movement efficiency of the motion, the greater difference of muscle synergy, and the more serious the torso compensation.

### 4.2. Motor Function Assessment in Stroke Patients

The correlation coefficients are shown in Table 2. All of the five features are significantly related with the FM score (*p* ≤ 0.001). The fitting chart between peak speed and torso balance degree with the FM score is shown in Figure 6 as an example. We also conduct the canonical correlation analysis to the five features and FM score and obtained correlation coefficient of 0.78. Clinically, the FM scale primarily assesses the independent joint motion of the upper limb but could not comprehensively evaluate the dyskinesia caused by hypertonia [39]. Compared with the FM scale, the evaluation features proposed in this paper can more effectively measure the upper limb motor dysfunction caused by dystonia, motor compensation, and abnormal muscle patterns.

To further verify the agreement between evaluation features and FM scale, the Bland–Altman plot was performed, shown as Figure 7. The presentation of the 95% limits of agreement (LoA) calculated as $\bar{d}\pm 1.96S_{d}$ is for visual judgement of how well two methods of measurement agree. In our results, almost all the points are within the 95% LoA, so the features have great consistency with the clinical FM scale.

## 5. Discussion

This study demonstrated that evaluation features extracted from kinematic and sEMG data can assess the upper limb motor function in stroke patients. These results can provide comprehensive descriptions of upward reaching movement and help to improve the personalized rehabilitation process.

### 5.1. Kinematic Data Analysis

With the development of the microsensor, the inertial sensor has been widely used in wearable devices in rehabilitation field. It has the advantages of low cost, small volume, low requirements for experimental environment, and convenient to use. The use of inertial sensors makes it possible to quantify the evaluation of motor function in motor cortical impairments patients, such as stroke. We can see from Figure 5 that the poststroke patients performed the reaching task at a small joint angle and speed, which is consistent with previous research [40, 41]. The joint angle denotes the motor ability, and the arm speed reflects the efficiency when completing a movement. Due to the loss of motor functional, the presence of weakness in stroke patients is reflected in these two features [42]. We observed in Figure 3 that the shoulder joint angle of severe subject (FM = 13) is not as smooth as subject from the mild-to-moderate (FM = 44) and control group. This indicates the arm tremble of severe patients when they complete the reaching task. Besides, in Figure 3, the abscissa value of inflection point in joint angle curve can also suggest the speed of the upper limb. The subject from the severe group takes longer time to lift his arm, which means lower in speed and agrees with values in Figure 5.

### 5.2. Muscle Synergy Analysis

For stroke patients, muscle synergy analysis is a useful method to identify abnormalities in muscle coordination. The altered structure of muscle synergy could reflect changes in neural excitability and affect the muscle coordination patterns. The NMF algorithm is used to extract muscle synergies from sEMG signals of multiple muscles. Tresch et al. found that the extracted synergies can reflect structures of the motor modules used by the motor system for movement control, rather than artefacts contingent upon the assumptions of NMF [43]. The factorization procedure essentially performs a dimensionality reduction by grouping the muscles that tend to covary in the dataset into individual synergies [25]. Evidence suggests that muscle synergy structure altered in stroke survivors from severe to mild impairment [17, 44].

In our previous study, alterations of synergies in subacute stroke patients were observed and the similarities compared with the control group were correlated with Brunnstrom stages [45]. In this paper, we also found that the muscle synergies altered in stroke patients with different FM scale as shown in Figure 4. We can see that in the first synergy from the severe group, the TRA is also coactivated with DELA and DELM, while the mild-to-moderate group is more similar to the control template. This may be due to the fact that stroke survivors in the severe group use shrugging shoulders as compensation strategy to assist with the reaching movement. The lack of TRI can be observed in both mild-to-moderate and severe groups, which may indicate that stroke patients cannot keep their upper arm straight well. Furthermore, researchers found that different subjects at different mechanical conditions use the same motor control strategies in cycling and stance [46, 47]. In our study, we found similar result that the muscle synergy within the control was relatively similar to each other, as the template shown in Figure 4.

### 5.3. Validation of Evaluation Features

Reaching is one of the effective skilled movements in human daily lives, and it needs to coordinate many muscles acting on related joints [48]. It is important to understand the motor control strategy and quantify the motor impairment level in reaching movement. To investigate the valid features, we also calculated the feature of normalized path length, trajectory accuracy, elbow joint angle, and move smoothness and other features during the reaching movement. Normalized path length is the ratio of real move path and reference path. Trajectory accuracy is the degree of deviation between patient motion trajectory and the real trajectory. Elbow joint angle is the motion range of elbow joint. Move smoothness is the jerk of the arm during the movement. However, these features have no significant relation to the FM score. Thus, they cannot be used as evaluation features. So, we selected the five features mentioned in the paper which can reflect the motor impairment level of stroke patients.

To prove the validity of the evaluation features, we calculate the Spearman correlation coefficients between fives features and FM scale and all the *p* values are ≤0.001 (Table 2). Taking the max shoulder angle feature as an example, in several patients, the max shoulder angle has weak correlation with the FM score while the others are highly correlated. Among which, three patients have different degrees of high muscle tension in clinical evaluation. These patients have a lower range of shoulder joint motion due to a decrease in joint mobility caused by excessive high muscle tension. However, the FM score of these three patients was not low; the reason is that the FM scale could not comprehensively evaluate the dyskinesia caused by hypertonia. There are two patients who achieved a greater range of shoulder motion during reaching movement due to the greater degree of torso compensation. Several patients complete the movement with the help of shoulder shrug compensation and also obtain a relatively large shoulder joint angle. These patients' trapezius muscle is activated abnormally due to the shrug compensation, so the muscle synergy similarity is relatively low.

### 5.4. Applications in the Field of Rehabilitation

Hemiplegia is one of the main symptoms of stroke or other spinal cord injury patients, which seriously affects patients' daily life and work. As the motor function of upper limbs is much more elaborate compared with lower limbs, no protocol proposed for the objective evaluation of the upper-extremities has achieved consensus [49]. Compared with the approaches of upper limb evaluation mentioned above, the five features we proposed can reflect the degree and efficiency of the completion of movement as well as muscle activity changes during the movement. This information is important for therapists to conduct personalized rehabilitation therapy for stroke patients. Thus, special training can be developed based on the results to make patients' features close to the control, for example, speed training and muscle strength training. More specifically, our model is a fusion of kinematics to and sEMG analysis that makes it possible for us to get a deeper understanding of human dynamic movement mechanism.

### 5.5. Limitations and Future Work

This study explored the evaluation features that can assess the motor function of stroke patients. The features we proposed combined the kinematic and sEMG data. However, the application of these features still has more work to do. First of all, poststroke duration may relate to FM score since the patients may receive a rehabilitation therapy or suffer motor function degeneration due to hemiplegia. Therefore, we recruited participants first attack receiving no therapy and with stroke duration no longer than 6 months to minimize the effect to our results. In future study, we should follow up specific stroke patients during recovery to investigate the influence of poststroke duration. Second, rehabilitation treatment the patient receives may affect the kinematic parameters and clinical scales. For example, robot-assisted training can lead to a significant reduction of motor impairment in subacute and chronic stroke patients by clinical outcome measures and kinematic parameters improvement [50]. We can study how the features change through treatment in the future. Finally, a comprehensive evaluation model based on these features should be established to grade the patients automatically in further studies. We should enlarge our dataset by containing more subjects and more experimental trials and realize the automatic grading by the classification algorithm. The model will provide great help for physicians to develop rehabilitation program for stroke patients.

## 6. Conclusions

In this paper, we mainly study a biomechanical evaluation method for upper limb motor function in stroke patients. We proposed five evaluation features based on kinematic and sEMG data to assess motor function of the upper limb in stroke patients. The five features of max shoulder joint angle, peak and average speeds, torso balance degree, and synergy similarity have significant difference in the stroke and control group and relatively high Spearman correlation coefficients with the FM scale. Furthermore, the Bland–Altman plots show a well consistency between the features and clinical FM scale. These features can provide not only motion descriptions but also kinetic basis of loss of motor function in stroke patients.

## Figures and Tables

**Figure 1:** Diagram of data collection. IMU and sEMG sensors are attached to the upper limb to collect kinematic and sEMG data during voluntary upward reaching. (a) Experimental setup and (b) the location of IMU and sEMG sensors.

**Figure 2:** Real-time shoulder angle of one subject from severe, mild-to-moderate, and control group separately. The severe patient has the narrowest joint angle and the lowest speed to reach the maximum of angle, and the mild-to-moderate patient is the next and then the control subject.

**Figure 3:** Number of synergies required to reconstruct muscle activation patterns in severe, mild-to-moderate, and control groups. Typically, 3 synergies were sufficient for all stroke and control groups.

**Figure 4:** Muscle synergy template of the control (a), mild-to-moderate (b), and severe (c) group. Three synergies are sufficient for subjects from three groups. Colorized bars show the relative weighting of a muscle and black bar with red represent group means and standard deviation.

**Figure 5:** Normalized feature values of in severe, mild-to-moderate, and control group (mean ± SEM). Significant differences exist between severe, mild-to-moderate, and control group (^∗^a significant difference; *p* ≤ 0.001).

**Figure 6:** The fitting chart of evaluation features and FM score. (a); (b) Features of peak speed and torso balance degree, respectively.

**Figure 7:** Bland–Altman plots showing the difference between evaluation features and FM scale against the mean of differences in upward reaching motion. Subplots (A)–(E) represent the Bland–Altman plot of max shoulder angle, peak speed, average speed, torso balance degree, and synergy similarity, respectively.

**Table 1:** General information of participants.

		Mean	SD	Range
Stroke group (*N* = 34)				
Severe impaired (*N* = 15)				
Age (year)		59.01	11.53	[44, 79]
Months since stroke		2.67	1.37	[0.83, 5.03]
Sex (male/female)	14/4			
Affected side (left/right)	13/5			
FM (out of 52)		18.67	12.97	[11, 28]

Mild-to-moderate impaired (*N* = 19)				
Age (year)		60.63	10.84	[38, 83]
Months since stroke		1.50	0.80	[0.60, 3.90]
Sex (male/female)	12/4			
Affected side (left/right)	6/10			
FM (out of 52)		41.38		[30, 51]

Control group (*N* = 25)				
Age (year)		59.16	9.97	[37, 77]
Sex (male/female)	13/12			

**Table 2:** Spearman's rank correlation coefficients between the features and the FM score.

Evaluation features	Correlation coefficient	*p*
Max shoulder angle	0.58	≤0.001
Peak speed	0.65	≤0.001
Average speed	0.62	≤0.001
Torso balance degree	−0.62	≤0.001
Synergy similarity	0.58	≤0.001

## Data Availability

The data used to support the findings of this study are available from the corresponding author upon request.
